The article "Dynamic Learning Rate in Deep CNN Model for Metastasis Detection and Classification of Histopathology Images" was published in 2021. Journal: Comput Math Methods Med.

# Dynamic Learning Rate in Deep CNN Model for Metastasis Detection and Classification of Histopathology Images

**DOI:** 10.1155/2021/5557168

**Published:** 2021-10-26

**Authors:** Anil Johny, K. N. Madhusoodanan

**Affiliations:** Department of Instrumentation, Cochin University of Science & Technology, Cochin, India

## Abstract

Diagnosis of different breast cancer stages using histopathology whole slide images (WSI) is the gold standard in determining the grade of tissue metastasis. Computer-aided diagnosis (CAD) assists medical experts as a second opinion tool in early detection to prevent further proliferation. The field of pathology has advanced so rapidly that it is possible to obtain high-quality images from glass slides. Patches from the region of interest in histopathology images are extracted and trained using artificial neural network models. The trained model primarily analyzes and predicts the histology images for the benign or malignant class to which it belongs. Classification of medical images focuses on the training of models with layers of abstraction to distinguish between these two classes with less false-positive rates. The learning rate is the crucial hyperparameter used during the training of deep convolutional neural networks (DCNN) to improve model accuracy. This work emphasizes the relevance of the dynamic learning rate than the fixed learning rate during the training of networks. The dynamic learning rate varies with preset conditions between the lower and upper boundaries and repeats at different iterations. The performance of the model thus improves and attains comparatively high accuracy with fewer iterations.

## 1. Introduction

Deep learning has emerged as a state-of-the-art technology in computer vision and speech recognition in recent years. The convolutional neural network (CNN) is the predominant method used in analyzing medical images [1]. CNN can learn spatial features in medical images adaptively using the backpropagation algorithm. Early diagnosis and treatment of breast cancer (BCa) prevents the proliferation of cells and thereby reduces morbidity and mortality [2]. In addition to diagnostic information, features such as nuclear atypia and the presence or absence of mitosis are indicative features indispensable for grading cancer stages. Metastasis detection with the assistance of the algorithm requires training the model with adequate images so that the model learns characteristic features in the spatial domain. Deep learning methods are effective [3] when the number of available images is large during the training stage. Model parameters and hyperparameters are selected foreseeing the application and availability of a sufficient number of images for training. The network then learns from the given dataset by updating the weights after each training step for the given number of classes and classifies images by reducing training loss. Optimization of the deep neural network (DNN) model involves fine-tuning of hyperparameters like the learning rate, batch size (BS), and momentum to improve model performance in task-specific applications. Conventional learning rate (LR) strategies include the constant learning rate, step decay, and exponential decay which possess a trial-and-error method to identify the optimal learning rate suited for the application. As a baseline method, model training with a fixed learning rate strategy is used than its counterparts. When the learning rate is too low, the model converges slowly, and for the high learning rate, the model training diverges resulting in suboptimal solutions. In optimal learning rate settings, the network converges after fewer iterations. The learning rate determines the extent of the loss gradient backpropagated in order to advance in the direction of global minima. If the gradient is stuck at local minima, noticeable progress is made only at the expense of computational cost. Adaptive LR methods for training involve the learning rate that changes by a predefined value, if no improvement is observed in accuracy after few epochs or stuck at local minima. On the other hand, in the nonadaptive schedule, the LR will either be constant till the end of the training or decrease gradually on every epoch by small steps. Other dynamic LR strategies that evolved recently are the cyclical learning rate (CLR) [4], stochastic gradient descent with warm restarts (SGDWR) [5] referred to as cosine annealing, and stochastic weight averaging (SWA) [6]. Variations in the learning rate are shown in Figure 1 for reference.

In the cyclical learning rate, the learning rate cyclically varies between the predefined lower and upper boundary values while training. Initially, the learning rate is kept very low which is then increased until it reaches the maximum value.

The learning rate then descends back to the initial value completing one cycle. Thus, a cycle consists of two steps with a fixed step size, which is the number of iterations over which the learning rate transitions from the minimum value to the maximum value. After every cycle of training, the pattern repeats itself till the last epoch in the triangular learning rate. Increasing the learning rate will have a short-term effect on accuracy, but in the long run, it alleviates loss during training.

In this work, we explore the optimal settings for attaining high classification accuracy for the CNN model by maneuvering the hyperparameter—learning rate. The dynamic learning rate is applied for the training phase which reduces the model loss significantly. During training, the optimizer uses the gradient descent algorithm to calculate the steepest descent and moves along the loss landscape in the direction opposite to the gradient at that point. The deep neural network with stochastic gradient descent (SGD) [7] is the training algorithm used for the training of deep neural networks. The optimizer updates the parameters (*θ*) after every epoch by *θ*_*t*_ = *θ*_*t*−1_ − *ϵ*_*t*_(*∂L*/*∂θ*), where *L* is the loss function, *ϵ*_*t*_ is the learning rate, and *θ*_*t*_ is the weights at time *t*. For low values of the learning rate, optimization takes place in small steps but convergence time increases at saddle point plateaus as shown in Figure 2. Increasing the learning rate is a fruitful way of escaping saddle points in nonconvex optimization problems. Cosine annealing is another modality of the dynamic learning rate schedule which starts with a large learning rate that is gradually decreased to a minimum value, then increased rapidly again, and the annealing schedule depends on the cosine function.

Equation (1) depicts the cosine annealing schedule:

(1) $$\begin{array}{c} \eta_{t}=\eta_{\min}^{i}+\frac{1}{2}\left(\eta_{\max}^{i}-\eta_{\min}^{i}\right)\left(1+\cos\left(\frac{T_{\text{cur}}}{T_{i}}\pi \right)\right). \end{array}$$

For the *i*-th run, the learning rate decays with cosine annealing for each batch as in Equation (1), where *η*_min_^*i*^ and *η*_max_^*i*^ are the ranges for learning rates and *T*_cur_ is the number of epochs elapsed since the last restart. Our aim is to explore optimum hyperparameter settings to attain CNN model performance with fewer epochs, where an aggressive annealing schedule is combined with periodic “restarts” to the original learning rate. The SWA algorithm for the learning rate [6] with default settings allows the learning rate to be controlled by an external learning rate scheduler or the default optimizer. In this strategy, the cyclic mode activates only after few epochs have elapsed. SWA will affect the final weights and the learning rate of the last epoch if batch normalization is also enabled during the model training.

The remaining section of the paper is organized as follows.  Section 2 outlines the related works. The dataset and evaluation metrics are described in Section 3.  Section 4 explains the typical CNN architecture.  Section 5 portrays the methodology followed in this work. Experimental results are drawn in Section 6. Discussion on the obtained results is included in Section 7.  Section 8 concludes with highlights and insights for further research.

## 2. Related Works

Detection of mitosis from breast cancer images is a challenging task since the slide has to be analyzed under a microscope by a pathologist which is tedious and often prone to subjective variations. Sommer et al. proposed a hierarchical learning workflow with a pixel-wise classifier [8] for automatic mitosis detection in breast cancer. Khan et al. [9] proposed a statistical approach which modeled the intensity of pixels in mitotic and nonmitotic regions by a gamma-Gaussian mixture model that effectively detects mitosis in standard histology images. Roullier et al. [10] presented a graph-based multiresolution approach for mitosis extraction in breast cancer histology images by segmentation at different resolutions based on a top-down approach. Fatakdawala et al. [11] in their work used an expectation-maximization-driven contour technique with overlap for segmentation of lymphocytes in histology images. Another similar method [12] for nucleus segmentation was based on multiscale Laplacian-of-Gaussian filtering performed after selecting the image foreground by graph-cut-based binarization. Irshad [13] aimed to improve the detection accurately by transforming color images into blue ratio image channels that better capture statistical and morphological features followed by binary thresholding and segmentation by refining the boundaries using an active contour model. Veta et al. [14] presented an automatic detection of mitotic cells in breast histology images by candidate extraction using a Chan-Vese level set, and classification was done by a statistical classifier trained with various features like shape, color, and texture. They also summarized various results from the Assessment of Mitosis Detection Algorithms (AMIDA) challenge [15] by multiple observers. Albayrak and Bilgin [16] proposed a Haralick feature descriptor with different window sizes to detect spatial dependency among different cellular structures in neighborhood pixels. They used machine learning to compare extracted features with various samples and suggested that an increase in window size improves accuracy in separating mitotic cells from nonmitotic cells. Machine learning (ML) algorithms are also applied to analyze handcrafted features in digital pathology images. Several preprocessing steps are carried out prior to applying ML algorithms. The extracted patches from whole slide images are then used for training traditional classifiers. Peikari et al. [17] used texture in the histology slide images that are identified by applying a Gaussian filter and calculated statistical measure from the histogram. They subsequently applied a support vector machine (SVM) classifier to distinguish clinically relevant regions. Machine learning techniques are widely used [18] nowadays in different medical images to leverage diagnosis and detection of several anomalies by analyzing the extracted handcrafted features. Similar attempts were also made by [19, 20] to train SVM classifiers based on features like nucleus properties, color, texture, and global image properties. These methods use handcrafted features with traditional classifiers which are inspired by domain-specific design and cannot handle the high variable sizes and shapes of mitoses very well.

The remarkable success of deep convolutional neural networks (CNN) in object detection and classification [21–24] of natural images inspired researchers to employ CNN in the analysis of medical images. Deep learning techniques extract global features from images which are subsequently used for classification of test images. Araújo et al. [25] performed training of the CNN model using patches and showed that when CNN is combined with the SVM algorithm, it yields better results. Spanhol et al. [26] used patches with different patch sizes (32 × 32, 64 × 64) using a sliding window scheme for training and classification of images. The reported accuracies were 83.3% for the patient level and 82.8% for the image level with a 200x magnification factor. Bejnordi et al. [27] compared performances of several algorithms and showed that deep learning with pretrained models outperformed in the machine learning challenge. Also, they revealed that the performance of few deep learning algorithms was comparable with expert pathologists interpreting WSI without time constraints. Cruz-Roa et al. [28] performed a deep learning approach in Invasive Ductal Carcinoma (IDC) using WSI of breast cancer and reported an F1-measure and balanced accuracy of 71.08% and 84.23%, respectively. In their work, the nonoverlapping patch size was 100 × 100 after discarding slide background images. The magnification independent method of training in [29] obtained an average recognition rate of 83.25% with a single-task CNN model and 82.13% in a multitask network. Litjens et al. [30] trained CNN with patch sizes of 128 × 128 under two different settings that obtained an area under the curve (AUC) between 0.88 and 0.90 for receiver operating characteristics (ROC). The pretrained model used by Chen et al. [31] trained 224 × 224 patches from WSI by image preprocessing and stain normalization steps and obtained an AUC score of 0.90. They also produced heat maps showing the probability of metastases in sentinel lymph nodes. An ensemble of deep learning networks by Kassani et al. [32] reported an accuracy of 90.84% for the single classifier and 94.64% for the ensemble method in the same open-access dataset. Wang et al. [33] utilized a 27-layer deep network to detect metastatic breast cancer in whole slide images of sentinel lymph nodes and won the Camelyon Grand Challenge 2016. Kieffer et al. [34] used possibilities of two pretrained models to train the dataset and compared performance before and after tuning. Yi et al. [35] used mammography data and a pretrained model for training, with hyperparameters for the model set to a dropout of 0.1, learning rate of 0.001, and batch size of 120 for 800 epochs. The GoogLeNet-based architecture produced a test accuracy of 85% among different algorithms. Sun et al. [36] used a probability map to delineate the tumor border using CNN trained from small patches cropped from histology images. Thagaard [37] presented an algorithm which can automatically detect cancer and classify WSI into metastasis subtypes in the Camelyon17 challenge which focused on patient-level analysis. From a large cohort of patients, they reached a weighted kappa value of 0.81 on the validation set. Xie et al. [38] used the BreakHis dataset for classifying histopathological images using pretrained models and obtained better results in binary as well as multiclass classification tasks. They also used the *K*-means clustering algorithm to cluster histopathology images to reduce interclass variation.

Motlagh et al. [39] compared the performance of pretrained Inception and ResNet models to identify subclasses of breast cancer and found that the latter was more sensitive to cancer datasets. They initialized the weight of their network by pretrained models and used the final layer for classifying cancer image datasets by updating continuously during each epoch. Deep neural network-based techniques suggested by Nahid et al. [40, 41] performed classification based on structural and statistical information from images using a combination of CNN and Long Short-Term Memory (LSTM). Patch-based classification was proposed by Roy et al. [42] using hierarchical CNN supported by data augmentation that produced a classification accuracy of 84.7% for the binary class. Jaiswal et al. [43] proposed a single-cycle learning rate policy with two steps throughout the training where LR increases in one step and decreases in the next iteration with a maximum learning rate of 0.00055 and a minimum of 0.0001. The method suggested by Pang et al. [44] takes input image slides of different resolutions scaled to256 × 256 on a pretrained model and reported 78.1% accuracy on embedding tile-based features. Fan et al. [45] generated a heat map using a pretrained model which is trained from patches cropped from whole slide images. Most works on CNN presented in the literature are based on pretrained models owing to ease of implementation and fewer epochs taken. On the other hand, Bardou et al. [46] created their own CNN model with 5 layers for binary and multiclass classification in their work along with a comparison of performance with traditional classifiers.

## 3. Dataset and Evaluation

The dataset PatchCamelyon (PCam) [47] is used in our work which contains 96 × 96 pixel color images (patches) annotated by experts with labels indicating the presence or absence of metastatic tissue. These patches were extracted from histopathology images of lymph node sections encompassing the benchmark classification dataset—PCam. Sample images from the database are shown in Figure 3. Evaluation metrics used in this work are precision, recall, and F1-score as in Table 1.

Each metric is calculated based on the true positive (TP), true negative (TN), false positive (FP), and false negative (FN) obtained from the confusion matrix at the end of training. The performance of the CNN model using the AUC metric shows the discriminative capability of the model on binary classification tasks.

The ROC curve is obtained by plotting the false-positive rate (FPR) and true-positive rate (TPR) at various thresholds. The area under the ROC curve is used to identify the capability of the model to differentiate benign and malignant classes which is crucial in diagnosing the disease. Optimizing the objective function in a deep neural network suffers from the existence of both local minima and global minima. Almost all local minima will have a very similar function value to the global minima, and hence, finding a local minimum is essential for model optimization by computing the gradient at every point. Such algorithms may get stuck at saddle points and never escape if the learning rate is less. Increasing the learning rate in this context has only short-term benefits. The cyclical learning rate is desirable in this scenario as it oscillates between two learning rate boundaries throughout the experiment.

Algorithm 1 shows the pseudocode for implementation of the cyclical learning rate and cosine learning rate. The mode select function accepts one strategy at a time, based on which the LR mode can be changed.  Algorithm 2 shows the pseudocode for implementing the stochastic weight averaging learning rate strategy.

## 4. CNN Architecture

The convolutional neural network is used to implement the proposed work.  Figure 4 shows the general architecture of a CNN which includes convolutional, pooling, flattening, and fully connected layers. The test image with different pixel intensities is given as input to the convolutional layer which consists of several filters to capture the main features in the image.

The pooling layer reduces the dimensionality of the features extracted by performing max pooling or average pooling. In max pooling, the maximum value is taken, whereas in average pooling, the average value will be considered in the filter region. The flattening layer converts the output of the previous layer into a one-dimensional array as the input of the fully connected layer. From the feature vector array, the fully connected layer performs classification and the result is given to the output layer. For binary classification, there will be two output classes, whereas for the multiclass classification task, there will be more than two outputs.  Algorithm 3 describes the pseudocode for the convolutional neural network.

CNN can capture important features automatically from the inputs, especially images when compared to multilayer perceptrons. The good performance and accuracy of CNN in image recognition applications [22] makes it more suitable than other traditional techniques. The challenge associated with CNN is that the number of images required for training the network is higher which results in more training steps. Moreover, hyperparameter tuning is inevitable for obtaining optimized performance results.

## 5. Methodology

The CNN model used for the experiment is a custom model with three convolutional layers with max pooling layers in between and ReLU [48] as the activation function after each convolutional layer.  Figure 5 shows the block diagram of the model used in our experiment. Details of model architecture are given in Table 2. Details of model configuration settings befitting our experiment are given in Table 3.  Algorithm 4 describes the pseudocode for the proposed CNN model.

In task-specific applications, there barely exists a definite method to find the number of layers or amount of neurons required in each layer for training the model. The selection of few parameters is based on our previous work in [49], and we found that the training to test the ratio of the dataset is fixed to 80 : 20 for a batch size of 32 with 500 epochs throughout the experiment. Initialization of the network weights is done using the Gaussian distribution with a low standard deviation for all the layers. The depth of deep learning and the number of neurons in each layer were selected after heuristic analysis since the size of the input image varies among different applications. In task-specific binary classification, in order to differentiate *benign* and *malignant* images in the test dataset, we chose binary cross-entropy (or log-loss) as a common practice to compute cross-entropy loss between true labels and predicted labels with the stochastic gradient descent optimization algorithm. The log-loss function for the binary class is represented in

(2) $$\begin{array}{c} \text{Loss}\left(L\right)=-\frac{1}{N}\overset{N}{\underset{i=1}{\sum }}y_{i}\cdot \log\left(p\left(y_{i}\right)\right)+\left(1-y_{i}\right)\cdot \log\left(1-p\left(y_{i}\right)\right), \end{array}$$

where *y* represents the ground truth label for the target binary class (label = 0 for benign, label = 1 for malignant) and *p*(*y*) is the probability of prediction of the sample being in that class for *N* images in the dataset. For each malignant image (*y* = 1), log(*p*(*y*)) is the log probability of it being malignant, and for each benign image, the log(1 − *p*(*y*)) component in the loss is the log probability for it being benign.

Training the neural networks with traditional learning methods, namely, exponential decay and step decay learning rate strategies, suffers from overfitting and longer convergence time due to the nonconvex nature of the loss landscape. Here, the training starts with a high learning rate, and towards the end of training epochs, LR decays monotonically till the last epoch in both methods. Towards the end of training, for small learning rates, the gradient enters local minima and never escapes [49].  Table 4 shows the obtained values of performance metrics corresponding to the conventional learning strategies mentioned in Section 1. By utilizing the dynamic nature of the learning rate during training, the gradient of the loss function is mitigated from being trapped at local minima or plateaus. For the current gradient vector and the learning rate, the gradient is recomputed after every iteration, and the process is repeated till it converges. The trained model is then used to predict the label for an unknown test image based on the loss function *L* as in Equation (2).

The changes in the learning rate from the default to cyclic mode [4] are done by changing the following parameters: lower limit (*base*_*lr*), upper limit (*max*_*lr*), and number of steps (*step*_*size*). These predefined parameters are activated along with the callback function during the training. In this mode, the learning rate increases from the lower limit in the cyclic mode with constant frequency but the amplitude is scaled after each cycle. The algorithm is shown in Figure 4. We selected the lower limit of *base*_*lr* = 0.001, upper limit of max_*lr* = 0.005, and step size *step*_*size* = 2500 in our experiment. The weights are updated after every epoch for each minibatch in the whole training data. Different modalities of CLR (*triangular*, *triangular2*, *exp*_*range*, and *custom cycle*) are applied subsequently for training the network. In the *triangular2* policy, the difference in lower and upper bounds is reduced to half after each cycle without affecting predefined learning rates. Another variation of triangular policy *exp*_*range* resembles *triangular2* but declines the cycle amplitude exponentially after each cycle which imparts controlled fine-tuning in *max*_*lr* during training. We also implemented the model with a *custom cycle* policy, a variant of the triangular method that scales the cycle amplitude sinusoidally. The accuracy values for each training phase are tabulated. After the training epochs, the model converges faster with competent classification performance as shown in Figure 6. The cosine annealing learning strategy is also applied to the same model to investigate the effect of warm restarts on training the model. Mode selection is done inside the callback function as mentioned in Algorithm 1 shown as Figure 4. The parameter *T*_max_ represents repetition cycles in the cosine annealing learning strategy, with restarts at the end of every cycle. The learning rate is varied in three ranges for each cycle under consideration. The *T*_max_ and LR range are set to different values as shown in Table 5 to estimate changes in performance in each case. We applied the stochastic weight averaging (SWA) method also in our model for training the dataset with batch normalization [52] in order to reduce covariate shift. The implementation algorithm is shown in Figure 5. The parameters in our method were set to change the LR after 75% of the epochs have been completed in both the *cyclic* and *constant* modes. Initial settings with a lower learning rate (lr = 0.001) enable the model to converge within a reasonable time. Furthermore, in high-dimensional weight space, local minima towards the end of every learning rate cycle accumulate near the boundary of the loss surface where the loss value is comparatively low [6]. By taking the average of several such points, it is possible to achieve a solution with a lower value of loss. The model is implemented with an SGD optimizer for computing the average of multiple points along its trajectory any time after 75% of total epochs have elapsed effectively making it an ensemble mode of training.

## 6. Results

The results obtained for each learning modality are tabulated and compared. The accuracy, precision, recall, F1-score, and AUC of the triangular learning rate are shown in Table 6. It reflects higher performance for all triangular learning strategies with *step*_*size* = 2500. Performance metrics for cosine annealing LR are given in Table 5 corresponding to various cycles. For each range of the learning rate, performance metrics obtained are shown. The performance of the native model for the SWA learning method is tabulated in Table 7.

The performance values for the CLR strategy are analyzed categorically. In the *triangular* method, the maximum accuracy is 91.84% while comparing all triangular LR methods with mean and median values of 91.4% and 91.2%, respectively. On the contrary, in the cosine annealing LR method, the maximum accuracy value is 91.8% for iteration with a cycle = 50 and a learning rate between 0.001 and 0.006.

When comparing the obtained values of performance metrics, it is evident that the model with a dynamic learning rate strategy outperforms the fixed learning rate. AUC for the fixed learning rate is obtained as 0.92, whereas a score greater than 0.97 is obtained for all dynamic learning rates which are considered. From the curves obtained, dynamic learning rates are found more suitable for the application considered.

Execution time and loss (*val*_*loss*) are two key factors which decide the efficiency of the algorithm on model training. The proposed model is implemented in Python3 using the Keras [53] library on a GPU-enabled Intel Core i7 processor-based system with 32 GB RAM.  Table 8 shows the average execution time required and validation loss for various dynamic learning strategies. The obtained results show that the triangular learning strategy generates minimum validation loss during training when compared to other learning strategies with a comparable time of execution. In general, we observed that all cyclical learning rates converge faster with few iterations and higher validation accuracy.

## 7. Discussion

For task-specific medical applications like the classification of histopathological images, we propose a custom model with a dynamic learning rate as it can be configured for the same. The cyclical learning rate shows better performance over the conventional learning rate. We experimented with both types of learning strategies on the model based on a common performance metric. All the performance metrics are equally considered in our experiment for analyzing the model predictability and trainability under different learning schemes. The fixed learning rate shows little improvement in accuracy after 50% of the epochs as shown in Figure 7, due to local minima while computing the cost gradient on the training dataset. On the other hand, significant improvement in model performance is obtained when the learning rate swings between the upper and lower learning ranges irrespective of the number of cycles. It is observed that the *triangular* learning policy produced the highest accuracy among the other CLR schemes as in Table 6. High precision and recall which are observed in the triangular cyclic method make it more suitable for the classification of histopathological images. In the case of the cosine learning rate, changing the upper and lower limits reflects in the model performance while keeping the number of cycles fixed as in Table 5. Accuracy is improved when the learning rate is between 0.001 and 0.0001 irrespective of the number of cycles. By changing the number of cycles per iteration and ranges of the learning rate, higher accuracy can be obtained in the SWA strategy. The performance metrics were calculated for constant and cyclic SWA learning strategies with and without batch normalization as shown in Table 5, where a notable performance metric is observed with batch normalization. This method utilizes the advantage of ensemble training where more than one neural network with different initializations averages the predictions from models to reduce the error rate. The performance of stochastic weight averaging with batch normalization in terms of accuracy is moderately high, but the capability of the model to differentiate binary class images is lesser than that of the triangular and cosine LR methods. From the results obtained in Section 5, it is apparent that triangular LR gives appreciable performance based on evaluation metrics.

## 8. Conclusion

A custom CNN model is designed and trained using a dynamic learning rate to improve the performance of the network for the classification of histology images. The learning rate is the crucial hyperparameter which decides the quality of CNN model training as it imparts fine-tuning in classification tasks. Using the standard database PCam, our custom model classified benign and malignant patches accurately by setting variable learning rates during the model training. We show that the use of cyclical learning rates for training produces promising optimal results than conventional learning rates. Changing the learning rate while training creates repercussions but benefits escaping from saddle points and local minima producing better accuracy. We conducted experiments for the accurate classification of histopathological images with various dynamic learning strategies. The performance of different methods is compared, and it is found that in applications which are task-specific, the triangular method outperforms other modalities in discriminating benign from malignant. Prediction of metastasis in medical images is effectuated with reduced false-positive rates. Training the CNN model with variable learning rates achieved 91.84% validation accuracy with lesser epochs than fixed learning rate counterparts. Increasing the learning rate during training assists the model to escape saddle points in the loss landscape and traverse towards global minima. By examining the area under the receiver operating characteristic curve for all learning modalities, dynamic learning rates produced superior classification accuracy in the detection of metastasized and benign cells in histopathology images.

## Figures and Tables

**Figure 1:** Different dynamic learning rate strategies. In both (a) and (b), the learning rate changes between the lower and upper boundaries and the pattern repeats till the final epoch.

**Figure 2:** Saddle point. Saddle points are pseudominima which represent neither local minima nor global minima in the loss landscape. The gradient is recomputed after every iteration till it converges.

**Figure 3:** Sample images from the database with ground truth labels. The label shows the presence of malignancy in two patches and absence in benign differentiated by the extent of staining in each image.

**Figure 4:** General architecture of CNN. The first convolutional layer extracts features from the input image with dimension *M* × *N* × *C* with *C* channels. The pooling layer performs dimensionality reduction, and the data is converted to a one-dimensional array by the flattening layer. The fully connected layer generates the output after classification.

**Figure 5:** Block diagram of the proposed model. Two fully connected dense layers in the model with sigmoid activation in the output layer perform the classification based on the features extracted by the previous convolutional layers.

**Figure 6:** Comparison of accuracy curves for different learning rates. The validation accuracy curves for all learning rate methods shown in the figure indicate a change in accuracy as epochs progress when compared with the fixed learning rate. Here, we observed that there is no noticeable change in validation accuracy for fixed LR where all other dynamic learning rates exhibit an appreciable increase in accuracy with epochs.

**Figure 7:** ROC curves. The figure depicts the highest AUC values obtained for various LR schemes during the experiment. The ROC curve of the model for different LR shows that it is able to discriminate malignant from benign.

**Algorithm 1:** Pseudocode for the cyclical learning rate (CLR).

**Algorithm 2:** Pseudocode for the stochastic weight averaging (SWA).

**Algorithm 3:** Pseudocode for the convolutional neural network.

**Algorithm 4:** Pseudocode for the proposed CNN model.

**Table 1:** Evaluation metrics used.

Metrics	Definition	Range
Accuracy	$\text{Acc}=\frac{\text{TP}+\text{TN}}{\text{TP}+\text{TN}+\text{FP}+\text{FN}}$	(0, 1)
Precision	Pr = TP/(TP + FP)	(0, 1)
Recall	*R* = TP/(TP + FN)	(0, 1)
F1-score	F1 = 2 × (Pr × Re/Pr + Re)	(0, 1)

**Table 2:** CNN model architecture details.

Layer	Dimension	Stride	Activation
Input	96 × 96 × 3	—	—
Convolutional layer	30@8 × 8	2	ReLU
Max pooling	3 × 3	1	—
Convolutional layer	100@5 × 5	2	ReLU
Max pooling	3 × 3	1	—
Convolutional layer	100@5 × 5	2	ReLU
Max pooling	3 × 3	1	—
Fully connected	300	—	ReLU
Fully connected	200	—	ReLU
Output	1	—	Sigmoid

**Table 3:** Overview of model configuration.

Model parameters and hyperparameters with ranges	
Model/hyperparameter	Value/range
Epochs [49]	500
Batch size [49]	32
Learning rate [49]	10^−2^–10^−4^
Optimizer [50, 51]	Stochastic gradient descent (SGD)
Loss function	Binary cross-entropy
Input shape	96 × 96
Pooling	Max pooling
Activation	ReLU

**Table 4:** Performance metrics for conventional learning strategies.

Learning method	Performance metrics				
	Accuracy	Precision	Recall	F1-score	AUC
Constant	0.8718	0.8561	0.8445	0.8535	0.92
Time based	0.8236	0.8258	0.8236	0.8233	0.91
Step decay	0.8173	0.8196	0.8173	0.8168	0.90
Exponential	0.8296	0.8317	0.8296	0.8293	0.91

**Table 5:** Cosine annealing (with restart) performance metric.

Learning rate	Accuracy	Precision	Recall	F1-score	AUC
Cosine LR (cycle = 10)					
0.01-0.001	0.8045	0.8446	0.8045	0.7983	0.94
0.01-0.0001	0.9068	0.9078	0.9069	0.9067	0.96
0.001-0.005	0.8861	0.8896	0.8858	0.8858	0.96
Cosine LR (cycle = 20)					
0.01-0.001	0.8361	0.8364	0.8361	0.8360	0.91
0.001-0.0001	0.8975	0.9020	0.8975	0.8971	0.97
0.001-0.005	0.8953	0.8955	0.8953	0.8953	0.96
Cosine LR (cycle = 50)					
0.01-0.001	0.8526	0.8652	0.8526	0.8512	0.95
0.001-0.0001	0.8714	0.8789	0.8713	0.8708	0.96
0.001-0.006	0.9183	0.9205	0.9183	0.9181	0.98
Cosine LR (cycle = 100)					
0.01-0.001	0.7866	0.8175	0.7866	0.7809	0.92
0.001-0.0001	0.9038	0.9072	0.9038	0.9036	0.97
0.001-0.006	0.68	0.7782	0.677	0.6433	0.88

**Table 6:** Cyclic learning rate (triangular) performance metric.

Learning strategy	Triangular LR (*step*_*size* = 2000)				
	Accuracy	Precision	Recall	F1-score	AUC
*triangular*	0.9184	0.9185	0.9183	0.9183	0.97
*triangular2*	0.9065	0.9066	0.9065	0.9064	0.97
*exp_range*	0.9116	0.9142	0.9116	0.9114	0.97
*custom cycle*	0.9048	0.9049	0.9048	0.9048	0.96

**Table 7:** Stochastic weight averaging (SWA) performance metric.

Learning method	SWA performance metric				
	Accuracy	Precision	Recall	F1-score	AUC
Constant	0.8892	0.8914	0.8892	0.8890	0.96
With BN	0.9001	0.9045	0.9001	0.8998	0.97
Cyclic	0.8236	0.8258	0.8236	0.8233	0.91
With BN (*f* = 5)	0.9105	0.9122	0.9105	0.9104	0.97

**Table 8:** Comparison of execution time and loss.

Learning strategy	Execution time (sec)	Validation loss
CLR (triangular learning strategies) (*step*_*size* = 2000)		
Triangular	19190.43	0.1996

SGDWR (cosine annealing strategies)		
cycle = 10	19064.76	0.2122
cycle = 20	18999.30	0.2765
cycle = 50	18998.74	0.2088
cycle = 100	18993.48	0.2303

SWA learning strategies		
Cyclic	19117.48	0.2609
Constant	18996.33	0.2369

Conventional learning strategies		
Fixed LR	19011.60	0.3298
Time-based decay	19001.54	0.3712
Step decay	19078.44	0.3891
Exponential decay	19057.34	0.3791

## Data Availability

The PCam dataset is used in the work, and it is available at the following link: https://github.com/basveeling/pcam.

## References

[1] Suzuki K. (2017). Overview of deep learning in medical imaging. *Radiological Physics and Technology*.

[2] Nahid A., Kong Y. (2017). Involvement of machine learning for breast cancer image classification: a survey. *Computational and Mathematical Methods in Medicine*.

[3] Shen D., Wu G., Suk H. I. (2017). Deep learning in medical image analysis. *Annual Review of Biomedical Engineering*.

[4] Smith L. N. Cyclical learning rates for training neural networks.

[5] Loshchilov I., Hutter F. SGDR: stochastic gradient descent with warm restarts. http://arxiv.org/abs/1608.03983.

[6] Izmailov P., Podoprikhin D., Garipov T., Vetrov D., Wilson A. G. (2019). Averaging weights leads to wider optima and better generalization.

[7] Bottou L. (2010). Large-scale machine learning with stochastic gradient descent.

[8] Sommer C., Fiaschi L., Hamprecht F. A., Gerlich D. W. Learning-based mitotic cell detection in histopathological images.

[9] Khan A. M., El-Daly H., Rajpoot N. M. A gamma-Gaussian mixture model for detection of mitotic cells in breast cancer histopathology images.

[10] Roullier V., Ta V., Lezoray O., Elmoataz A. Graph-based multi-resolution segmentation of histological whole slide images.

[11] Fatakdawala H., Jun Xu, Basavanhally A. (2010). Expectation–maximization-driven geodesic active contour with overlap resolution (EMaGACOR): application to lymphocyte segmentation on breast cancer histopathology. *IEEE Transactions on Biomedical Engineering*.

[12] al-Kofahi Y., Lassoued W., Lee W., Roysam B. (2010). Improved automatic detection and segmentation of cell nuclei in histopathology images. *IEEE Transactions on Biomedical Engineering*.

[13] Irshad H. (2013). Automated mitosis detection in histopathology using morphological and multi-channel statistics features. *Journal of Pathology Informatics*.

[14] Veta M., van Diest P. J., Pluim J. P. W., Gurcan M. N., Madabhushi A. (2013). Detecting mitotic figures in breast cancer histopathology images. *Medical Imaging 2013: Digital Pathology*.

[15] Veta M., van Diest P. J., Willems S. M. (2015). Assessment of algorithms for mitosis detection in breast cancer histopathology images. *Medical Image Analysis*.

[16] Albayrak A., Bilgin G., Vuksanovic B., Zhou J., Verikas A. (2013). Breast cancer mitosis detection in histopathological images with spatial feature extraction.

[17] Peikari M., Gangeh M. J., Zubovits J., Clarke G., Martel A. L. (2016). Triaging diagnostically relevant regions from pathology whole slides of breast cancer: a texture based approach. *IEEE Transactions on Medical Imaging*.

[18] Komura D., Ishikawa S. (2018). Machine learning methods for histopathological image analysis. *Computational and Structural Biotechnology Journal*.

[19] Han J. W., Breckon T. P., Randell D. A., Landini G. (2012). The application of support vector machine classification to detect cell nuclei for automated microscopy. *Machine Vision and Applications*.

[20] Fondón I., Sarmiento A., García A. I. (2018). Automatic classification of tissue malignancy for breast carcinoma diagnosis. *Computers in Biology and Medicine*.

[21] Krizhevsky A. (2009). Learning multiple layers of features from tiny images.

[22] Krizhevsky A., Sutskever I., Hinton G. E. (2017). ImageNet classification with deep convolutional neural networks. *Communications of the ACM*.

[23] Szegedy C., Liu W., Jia Y. Going deeper with convolutions.

[24] Szegedy C., Vanhoucke V., Ioffe S., Shlens J., Wojna Z. Rethinking the inception architecture for computer vision.

[25] Araújo T., Aresta G., Castro E. (2017). Classification of breast cancer histology images using convolutional neural networks. *PLoS One*.

[26] Spanhol F. A., Oliveira L. S., Petitjean C., Heutte L. Breast cancer histopathological image classification using convolutional neural networks.

[27] Ehteshami Bejnordi B., Veta M., Johannes van Diest P. (2017). Diagnostic assessment of deep learning algorithms for detection of lymph node metastases in women with breast cancer. *JAMA*.

[28] Cruz-Roa A., Basavanhally A., Gonzalez F., Gurcan M. N., Madabhushi A. (2014). Automatic detection of invasive ductal carcinoma in whole slide images with convolutional neural networks. *Medical Imaging 2014: Digital Pathology*.

[29] Bayramoglu N., Kannala J., Heikkila J. Deep learning for magnification independent breast cancer histopathology image classification.

[30] Litjens G., Sánchez C. I., Timofeeva N. (2016). Deep learning as a tool for increased accuracy and efficiency of histopathological diagnosis. *Scientific Reports*.

[31] Chen R., Jing Y., Jackson H. (2016). Identifying metastases in sentinel lymph nodes with deep convolutional neural networks. https://arxiv.org/abs/1608.01658.

[32] Kassani S. H., Kassani P. H., Wesolowski M., Schneider K. A., Deters R. (2019). Classification of histopathological biopsy images using ensemble of deep learning networks.

[33] Wang D., Khosla A., Gargeya R., Irshad H., Beck A. H. (2016). Deep learning for identifying metastatic breast cancer.

[34] Kieffer B., Babaie M., Kalra S., Tizhoosh H. Convolutional neural networks for histopathology image classification: training vs. using pre-trained networks.

[35] Yi D., Sawyer R. L., Au D. C. I. (2017). Optimizing and visualizing deep learning for benign/malignant classification in breast tumors.

[36] Sun Y., Xu Z., Strell C. Detection of breast tumour tissue regions in histopathological images using convolutional neural networks.

[37] Thagaard J. (2017). Detecting lymph node metastases in breast cancer using deep learning.

[38] Xie J., Liu R., Luttrell J., Zhang C. (2019). Deep learning based analysis of histopathological images of breast cancer. *Frontiers in Genetics*.

[39] Motlagh M. H., Jannesari M., Aboulkheyr H. (2018). Breast cancer histopathological image classification: a deep learning approach.

[40] Nahid A. A., Mehrabi M. A., Kong Y. (2018). Histopathological breast cancer image classification by deep neural network techniques guided by local clustering. *BioMed Research International*.

[41] Nahid A., Kong Y. (2018). Histopathological breast image classification using local and frequency domains by convolutional neural network. *Information*.

[42] Roy K., Banik D., Bhattacharjee D., Nasipuri M. (2019). Patch-based system for classification of breast histology images using deep learning. *Computerized Medical Imaging and Graphics*.

[43] Jaiswal A. K., Panshin I., Shulkin D., Aneja N., Abramov S. (2019). Semi-supervised learning for cancer detection of lymph node metastases.

[44] Pang H., Lin W., Wang C., Zhao C. Using transfer learning to detect breast cancer without network training.

[45] Fan K., Wen S., Deng Z. (2019). Deep learning for detecting breast cancer metastases on WSI. *Innovation in Medicine and Healthcare Systems and Multimedia*.

[46] Bardou D., Zhang K., Ahmad S. M. (2018). Classification of breast cancer based on histology images using convolutional neural networks. *IEEE Access*.

[47] Veeling B. S., Linmans J., Winkens J., Cohen T., Welling M. (2018). Rotation equivariant CNNs for digital pathology.

[48] Agarap A. F. (2019). Deep learning using rectified linear units (ReLU). https://arxiv.org/abs/1803.08375v2.

[49] Johny A., Madhusoodanan K. N., Nallikuzhy D. T. J. (2020). Optimization of CNN model with hyper parameter tuning for enhancing sturdiness in classification of histopathological images. *SSRN Electronic Journal*.

[50] Breuel T. M. (2015). The effects of hyperparameters on SGD training of neural networks. http://arxiv.org/abs/1508.02788.

[51] Ruder S. (2017). An overview of gradient descent optimization algorithms. https://arxiv.org/abs/1609.04747.

[52] Ioffe S., Szegedy C. (2015). Batch normalization: accelerating deep network training by reducing internal covariate shift.

[53] Chollet F. (2015). Keras. https://keras.io.

